# Curative Effects of Remote Home Management Combined with Feng's Spinal Manipulation on the Treatment of Elderly Patients with Lumbar Disc Herniation

**DOI:** 10.1155/2022/1420392

**Published:** 2022-01-25

**Authors:** Yaqing Min, Peng Xu

**Affiliations:** ^1^Pla Spine Center of Manipulative Orthopedics, Air Force Medical Center, Pla 100142, Beijing, China; ^2^Department of Rehabilitation Medicine, Baotou Mongolian Traditional Chinese Medicine Hospital, Baotou 014040, Inner Mongolia Autonomous Region, China

## Abstract

**Objective:**

To explore the curative effects of remote home management combined with Feng's spinal manipulation on the treatment of elderly patients with lumbar disc herniation (LDH).

**Methods:**

The clinical data of 100 patients with LDH in our hospital (December 2019–December 2020) were retrospectively reviewed. The 100 patients were equally divided into a routine treatment group and interventional group according to the order of admission. The routine treatment group received conventional rehabilitation training, and the interventional group received remote home management combined with Feng's spinal manipulation. The Oswestry disability index (ODI) and straight leg raising test were adopted for the assessment of the degrees of dysfunction and straight leg raising angles of the two groups after intervention. The curative effects of the two rehabilitation programs were evaluated.

**Results:**

Compared with the routine treatment group, the interventional group had a remarkably higher excellent and good rate (*P* < 0.05), a significantly lower average ODI score after intervention (*P* < 0.001), notably higher straight leg raising angle, surface AEMG (average electromyogram) during stretching and tenderness threshold after intervention (*P* < 0.001), markedly lower muscular tension, surface AEMG during buckling, and flexion-extension relaxation ratio (FRR; (*P* < 0.001)), and much higher quality of life scores after intervention (*P* < 0.001).

**Conclusion:**

The remote home management combined with Feng's spinal manipulation, as a reliable method to improve the quality of life and the back muscular strength of the elderly patients with LDH, can substantially increase the straight leg raising angle and reduce the degree of dysfunction. Further study is conducive to establishing a better solution for the patients with LDH.

## 1. Introduction

Lumbar disc herniation (LDH) is a common chronic orthopedic disease, with acute lumbar muscle sprain, excessive weight, lumbar spondylolisthesis, spinal stenosis, etc. Being the inducing factors. Although LDH does not affect the patients' life safety [1], the dysfunction and the changes of waist shape caused by this disease oppress and damage the nerve of cauda equina, which results in limb numbness and pain and even incontinence or paraplegia in severe cases [2]. As the living standard and socioeconomic level improve and the pace of life accelerates, the incidence of LDH is increasing year by year. Accordingly, people have begun to pay more attention to the prevention and rehabilitation of LDH [3, 4]. In Western medicine, the patients with LDH are treated with oral medicine and external application. If their conditions aggravate at the middle and later stages of the disease, lumbar discectomy and ozone injection will be performed. However, these treatments have unsatisfactory curative effects, high risk, and great trauma to the body and easily cause complications [5, 6]. Feng's spinal manipulation adopts spinal fixed-point rotation reduction to correct the vertebral displacement, and its curative effects have been confirmed in the treatment of sequestered LDH [7]. Remote home management uses WeChat to establish communication between doctors and patients, which breaks time and space limits and is efficient, convenient, and interactive. Its effects have been confirmed in the perioperative period nursing for the patients with coronary heart disease treated by percutaneous coronary intervention [8]. Currently, there are no studies confirming the treatment effect of remote home management combined with Feng's spinal manipulation for elderly patients with LDH. Based on the previous clinical treatment experience, this study implemented the combination therapy for elderly patients with LDH, aiming at providing effective rehabilitation programs for these patients, with the results reported as follows.

## 2. Materials and Methods

### 2.1. General Data

The clinical data of 100 patients with LDH in our hospital (December 2019–December 2020) were retrospectively reviewed. The 100 patients were divided into a routine treatment group and interventional group according to the order of admission, with 50 patients in each group. The study was performed in accordance with the Declaration of Helsinki (2013) [9].

### 2.2. Inclusion and Exclusion Criteria

#### 2.2.1. Inclusion Criteria

① The patients met the diagnostic criteria for this disease in *Lumbar Disc Herniation* [10], and their diagnoses were confirmed by CT (Computed Tomography) and MRI (Magnetic Resonance Imaging). The patients had the clinical symptoms of lumbago, sciatica, radiating pain in lower limbs, myasthenia, and so on; ② the patients lost lumbar lordosis and had lumbar scoliosis; ③ the patients were ≥60 years old, and they tested positive in the straight leg raising test and augmentation test; and ④ the patients had dysesthesia or muscular atrophy in the affected innervating areas.

#### 2.2.2. Exclusion Criteria

① The patients had lumbar spondylolisthesis or spinal stenosis; ② the patients were complicated with severe osteoporosis or lumbar trauma; ③ the patients suffered from the cerebral, cardiac, renal, or hematopoietic system dysfunction; and ④ there was skin ulceration or infection around the lesion sites.

### 2.3. Methods

The routine treatment group received conventional rehabilitation training. ① In the first stage, the patients took supine position, straightened one leg, flexed the knee and hip of the other leg, held the flexed knee with both hands, and pulled towards the chest and alternated legs. Then, the patients took prone position and raised the two legs by turns, with the knees keeping straight. Each exercise was held for 3–5 s and performed 30 times a day. ② In the second stage, the patients laid flat on a hard bed board and were supported by the head, elbows, and feet. The patients raised the hips as high as possible, held up the whole body with the hands and feet, and stretched the head and limbs back, with the abdomen flattening against the bed and acting as a flying swallow. Each exercise was held for 8–10 s and performed 40 times a day. ③ In the third stage, the patients took supine position, flexed both knees, elevated the pelvis, pressed both hands under the buttocks, and raised the lower limbs, with the feet and back as the supporting points. In addition, the patients took standing position, put one leg on the back of a chair, leaned forward to press the leg, and alternated the legs. Each exercise was held for 8–10 s and performed 30 times a day. ④ In the forth stage, the patients were guided to properly use the belt to avoid spine injury caused by activities [11, 12].

The interventional group received the remote home management combined with Feng's spinal manipulation, with the specific implementation step as follows.

#### 2.3.1. Remote Home Management

① Home nursing teams were established, and the main members were resident doctors, head nurses, responsible leaders, and primary nurses. Relevant knowledge training was carried out for them. ② One day before discharge, the primary nurses conducted discharged health education on the patients and set up patient files after collecting relative information through the questionnaire. Also, the primary nurses discharged Home Nursing and Rehabilitation Manual for Patients with LDH and the table of home-nursing rehabilitation training path to the patients. ③ WeChat groups were set up, and each patient was required to take a video of functional exercise and upload it to the WeChat group every week, which played the role of supervision in the gap of home visits. ④ After the patients being discharged, the duty nurses conducted regular family follow-up visits and rehabilitation training guidance to the LDH patients according to the contents of home-nursing rehabilitation training path. ⑤ Before the follow-up, the primary nurses should contact the patients in advance. The specific follow-up time depended on the specific circumstances of the patient and was usually 30–60 minutes. During the follow-up, the patients' disease conditions and functional exercise situations were assessed, and they were given targeted health education according to the existing nursing problems. ⑥ After the follow-up, the primary nurses filled in the tracking table of home nursing.

#### 2.3.2. Feng's Spinal Manipulation

The patient took the sitting position. The doctor extended the right hand forward from the patient' right armpit, and pressed the right palms on the patient' left shoulder. At the same time, the doctor should repeatedly advise the patient to put both feet on the ground and not to move the buttocks (the assistant stood facing the patient with both legs clamping around the patient's left thigh and with both hands pressing against the patient's left groin, to ensure the patient sits upright). The doctor used the left thumb to hold against the patient's right side of the deviated spinous processes and pulled the patient's left shoulder with the right hand to make the patient's body bend forward 20–50° and then bend right, better >45°. When the patient reached the maximum lateral bending position, the doctor used his/her right upper limb to make the patient's body horizontally rotate to the posteromedial. At the same time, the doctor's left thumb pushed against the vertebral spinous process towards the upper left. At this time, the doctor could hear the sound of embolia and felt the vertebral displacement. After that, the doctor moved booth thumbs from up to down to smooth the supraspinous ligaments and loosen the psoas muscles. Finally, the doctor used a thumb to press the spinous processes one by one from up to down to examine whether the deviated spinous processes were set right and whether the interspinous gaps had equal width. The manual reduction was conducted on alternate days. Patients in the two groups received intervention for 3 months.

### 2.4. Observational Indexes

The modified Macnab evaluation standard [13] was adopted to appraise the intervention effects of the two groups. If the symptoms completely disappeared and the patients returned to normal life and work, the curative effects were considered excellent; if the patients had mild symptoms and slightly limited activities, which did not affect the normal work and life, the curative effects were considered good; if the clinical symptoms were alleviated after intervention, but the daily activities were limited and affected the normal work and life, the curative effects were considered fair; and if the symptoms were not alleviated and even aggravated after intervention, the curative effects were considered poor. Good rate = (number of excellent cases + number of fair cases)/total number of cases × 100%.

The Oswestry disability index [14] (ODI) was adopted for the assessment of the degrees of dysfunction of the two groups after intervention. This scale consisted of 10 questions, including lifting, walking, standing, pain intensity, sleeping, sex life, social life, personal care, sitting, and travelling. Each question had 6 options, with the score from 0 point to 5 points, and the total score was 50 points. ODI = actual score/50 × 100% (for the patients who answered all the questions). ODI = actual score/45 × 100% (for the patients who only answered 9 questions). Higher scores indicated severer dysfunction.

In the straight leg raising test, the patient took supine position and both legs straightened naturally. The examiner held the patient's ankle with one hand and put the other hand above the knee joint so that the knee joint kept upright and rose to a certain angle. When the patients felt radiating pain or numbness in lower limbs, or the original pain or numbness increased, they tested positive [15]. A digital angle finder (manufacturer: Shanghai Grows Instrument Co., Ltd.) was adopted to record the raising angles.

The mechanical effects of lumbar muscle after intervention were compared between the two groups. The OE-220 muscular tension/tenderness detector (manufacturer: Japan Ito Manufacturing Vietnam Co., Ltd.) and MyoNet-AOW surface electromyography feedback machine (manufacturer: Shanghai Nuocheng Electric Co., Ltd.) were adopted to detect the surface AEMG (average electromyography) during stretching, AEMG during buckling, muscular tension, and tenderness threshold. Flexion-extension relaxation ratio (FRR) = surface AEMG during buckling/surface AEMG during stretching.

The 36-item short-form health survey questionnaire (SF-36) [16] was adopted for the evaluation of the living quality of the two groups after 4 weeks of intervention. This questionnaire included somatic role, emotional role, physical function, general health, social function, mental health, and vitality, with an aggregate score of 100 points for each dimension. The reliability coefficient of each dimension was ≥0.7, indicating a good internal consistency of the scale. Higher scores indicated better quality of life of patients.

### 2.5. Statistical Treatment

The professional statistical software SPSS23.0 was adopted for data processing, and GraphPad Prism 7 (GraphPad Software, San Diego, USA) was used to draw graphs of the data in this study. The count data were tested by *X*^2^ and expressed by [*n*(%)]. The measurement data were tested by *t* and expressed by mean ± SD. When *P* < 0.05, the differences were considered statistically significant.

## 3. Results

### 3.1. Comparison of Clinical Data

No notable difference in sex ratio, mean age, mean duration of disease, place of residence, and other clinical data was observed between the two groups (*P* > 0.05), which were comparable, as illustrated in Table 1.

### 3.2. Comparison of Curative Effects

Compared with the routine treatment group, the excellent and good rate in the interventional group was remarkably higher (*P* < 0.05; Table 2).

### 3.3. Comparison of ODI Scores

Compared with the routine treatment group, the average ODI score of the interventional group after intervention was much lower (*P* < 0.001; Figure 1).

### 3.4. Comparison of Straight Leg Raising Angles

Compared with the routine treatment group, the straight leg raising angle of the interventional group after intervention was notably higher (*P* < 0.001; Figure 2).

### 3.5. Comparison of the Mechanical Effects of Lumbar Muscle

Compared with the routine treatment group, the surface AEMG during stretching and tenderness threshold of the interventional group after intervention were notably higher (*P* < 0.001), but the muscular tension, surface AEMG during buckling, and FRR of the interventional group after intervention were markedly lower (*P* < 0.001), as shown in Table 3.

### 3.6. Comparison of Quality of Life Scores

Compared with the routine treatment group, the quality of life scores in the interventional group after intervention were all notably higher (*P* < 0.001; Table 4).

## 4. Discussion

According to modern medicine [17], the lumbar disc degeneration or trauma causes the nucleus pulposus and annulus fibrosus to protrude towards the spinal canal and to constrict the spinal cord or nerve root, which leads to LDH, the inflammatory changes of local hyperemia, and edema. The posterior longitudinal ligaments of the lumbar segment are narrower in the intervertebral disc plane, whose two sides are not covered by ligaments, and the posterior lateral side of the annulus fibrosus is narrower, so the disc herniation mostly occurs in the posterior lateral side. Because the posterior longitudinal ligaments can strengthen the annulus fibrosus, disc herniation less occurs in the midline [18]. LDH decreases relaxation of the ligaments around the lesion sites and increases the instability of the lumbar vertebrae. The herniated intervertebral discs compress the nerves, leading to lumbar and leg pain and lumbar hypofunction and even loss of living ability in severe cases. Currently, the major treatment for LDH is orally taking nonsteroidal anti-inflammatory drugs and hormone drugs. Although these drugs can effectively alleviate the patients' symptoms, long-term use would produce gastrointestinal adverse reactions and the patients are at a risk of recurrence after drug withdrawal [19]. The rehabilitation training, targeting at the specific disease conditions of the patients, exercises their lumbar muscle function. The training can maintain the stability of the lumbar vertebrae, accelerate local blood circulation, restore nerve function, and speed up the patients' recovery. However, the single rehabilitation training has a long treatment cycle and is likely to trigger adverse emotions from the patients, resulting in poor treatment compliance.

With the wide application of Internet technology, remote home management, as the improvement and supplement to the continuous nursing service, provides the patients with nursing services through the transmission, management, and coordination of information technology (WeChat) in practice, and with professional and personalized guidance by the aid of the effective, timely, and updated information transmission and the two-way communication and exchange. The remote home management can effectively break the limitations of space and offer the patients better nursing after discharge [20], with the effect that has been proven in elderly patients who received cardiac pacemaker implantation [21]. Feng's spinal manipulation, taking “joint semidislocation and sinews off-position” as its theoretical basis, adopts the spinal fixed-point rotation reduction to quickly correct the vertebral displacement, relieve the synovium incarceration, restore the mechanical balance of the lumbar vertebrae, and improve blood circulation of regional tissue. Therefore, Feng's spinal manipulation can speed up the patients' recovery, and its curative effects have been confirmed in the treatment of acute lumbar muscle sprain [22]. This study implemented the remote home management combined with Feng's spinal manipulation on the treatment of elderly patients with LDH, and with the help of the WeChat platform that has the characteristics such as simple operation, remote home management can break through the limitation of time and space, which facilitates the daily communication between healthcare workers and patients, thereby ensuring the information effectiveness. Compared with the routine treatment group, patients in the interventional group achieved remarkably higher surface AEMG during stretching and tenderness threshold after intervention (*P* < 0.001) and markedly lower muscular tension, surface AEMG during buckling, and FRR (*P* < 0.001), which showed that the remote home management combined with Feng's spinal manipulation helped to relieve the patients' pain and restore their lumbar function. The action mechanism of Feng's spinal manipulation was speculated as follows: ① Bones, muscles, and joints performed passive movements under Feng's spinal manipulation, which acted as a booster pump and promoted general blood circulation. ② Feng's spinal manipulation could restore the dislocated and disordered joints to the normal physical locations by promoting the movements of these joints and spasmodic muscles, which could effectively relieve joint incarceration and improve lumbar dysfunction. ③ The manipulation also helped to reopen the soft tissue (such as adhesive ligaments and muscles) and restore the muscle elasticity besides promoting the movements of bones and joints [23, 24]. The straight leg raising test, as a common examining method, could reflect the severity of sciatica and LDH and the compression of nerve root [25]. This study adopted straight leg raising test to evaluate the curative effects of the two groups after intervention. The straight leg raising angle of the interventional group was notably higher compared with the routine treatment group (*P* < 0.001), indicating that the joint intervention could effectively ease the patients' lumbocrural pain and substantially improve their movement disorders. The joint intervention had obviously better curative effects than the conventional rehabilitation treatment.

The limitations of the study were as follows. Firstly, the samples selected in the study were only the local patients and did not include the patients from other regions, so the results might be influenced by the small sample size and regional culture. Besides, the long-term effects should be considered in the actual treatment for LDH because it is a recurrent chronic disease. However, the study did not carry out the follow-up visit for a long term due to the limited time. Finally, the study adopted the straight leg raising test, mechanical effects of lumbar muscles, and other observed indexes. The clinical objective indexes such as the hematology and electromyography can be added when the experimental conditions allow.

## Figures and Tables

**Figure 1:** Comparison of ODI scores after intervention. *Note*. The abscissa indicates the routine treatment group and the interventional group, and the ordinate indicates the ODI score (points); the average ODI scores of the routine treatment group and the interventional group after intervention were (32.68 ± 2.43) points and (21.02 ± 2.84) points, respectively;  ^*∗*^a remarkable difference in the average ODI scores between the two groups after intervention (*t* = 22.059, *P* < 0.001).

**Figure 2:** Comparison of the straight leg raising angles after intervention. *Note*. The abscissa indicates the routine treatment group and the interventional group, and the ordinate indicates the straight leg raising angle (°); the straight leg raising angles of the routine treatment group and the interventional group after intervention were (71.32 ± 2.75) and (61.94 ± 1.48), respectively;  ^*∗*^ a notable difference in the straight leg raising angles between the two groups after intervention (*t* = 21.238, *P* < 0.001).

**Table 1:** Comparison of clinical data (*n* = 50).

Item	Routine treatment group	Interventional group	*X* ^2^/*t*	*P*
Sex			0.367	0.545
Male/female	27/23	30/20		
Body mass index (mean ± SD, kg/m^2^)	22.37 ± 0.73	22.45 ± 0.69	0.563	0.575
Mean age (mean ± SD, years)	69.90 ± 4.38	69.42 ± 4.22	0.558	0.578
Mean duration of disease (mean ± SD, months)	34.94 ± 4.61	36.04 ± 5.19	1.120	0.265
Modified Japanese Orthopaedic Association (M-JOA) score before intervention (mean ± SD, points)	6.82 ± 1.56	6.36 ± 1.83	1.353	0.179
Comparison of the LDH segments			0.174	0.677
L4-5	33 (66.00)	31 (62.00)		
L5-S1	17 (34.00)	19 (38.00)		
Straight leg raising angle (mean ± SD, °)	53.69 ± 2.02	53.88 ± 2.30	0.439	0.662
Education level				
University/college	3 (6.00)	4 (8.00)	0.154	0.695
Middle school	17 (34.00)	14 (28.00)	0.421	0.517
Primary school	30 (60.00)	32 (64.00)	0.170	0.680
Place of residence			0.170	0.680
Urban areas	32 (64.00)	30 (60.00)		
Rural areas	18 (36.00)	20 (40.00)		

**Table 2:** Comparison of curative effects [*n*(%)].

Group	*n*	Excellent	Good	Fair	Poor	Excellent and good rate
Interventional group	50	17 (34.00)	30 (60.00)	3 (6.00)	0 (0.00)	94.00 (47/50)
Routine treatment group	50	12 (24.00)	27 (54.00)	9 (18.00)	2 (4.00)	78.00 (39/50)
*X* ^2^						5.316
*P*						<0.05

**Table 3:** Comparison of the mechanical effects of lumbar muscle.

Group	*n*	Surface AEMG during stretching (*μ*V)	Muscular tension (N)	Tenderness threshold (%)	Surface AEMG during buckling (*μ*V)	FRR
Interventional group	50	105.99 ± 4.88	45.26 ± 1.73	95.56 ± 3.89	62.24 ± 2.43	0.51 ± 0.04
Routine treatment group	50	93.90 ± 2.76	54.81 ± 2.49	84.97 ± 2.17	72.18 ± 1.30	0.70 ± 0.04
*t*		15.248	22.272	16.811	25.504	23.750
*P*		<0.001	<0.001	<0.001	<0.001	<0.001

**Table 4:** Comparison of quality of life scores.

Group	n	Somatic role	Emotional role	Physical function	Social function	General health	Physical pain	Vitality	Mental health
Interventional group	50	80.08 ± 2.88	81.38 ± 4.25	77.84 ± 3.78	73.30 ± 3.25	76.56 ± 3.67	76.92 ± 4.69	72.54 ± 5.33	78.14 ± 3.52
Routine treatment group	50	71.46 ± 4.09	70.42 ± 4.66	69.50 ± 3.29	66.78 ± 2.82	70.56 ± 3.72	62.64 ± 2.85	61.14 ± 4.19	72.40 ± 2.27
*t*		12.185	12.288	11.768	10.715	8.119	18.399	11.890	9.690
*P*		<0.001	<0.001	<0.001	<0.001	<0.001	<0.001	<0.001	<0.001

## Data Availability

Data used to support the findings of this study are available on reasonable request from the corresponding author.

## References

[1] Wang Z., Chen Z., Wu H. (2020). Treatment of high-iliac-crest L5-S1 lumbar disc herniation via a transverse process endoscopic transforaminal approach. *Clinical Neurology and Neurosurgery*.

[2] Xu J., Ding X., Wu J. (2020). A randomized controlled study for the treatment of middle-aged and old-aged lumbar disc herniation by Shis spine balance manipulation combined with bone and muscle guidance. *Medicine*.

[3] Wu X., Ma Y., Ding R., Xiao X., Yang D. (2021). Should adjacent asymptomatic lumbar disc herniation be simultaneously rectified? a retrospective cohort study of 371 cases that received an open fusion or endoscopic discectomy only on symptomatic segments. *The Spine Journal*.

[4] Yang X., Li F., Xin D. (2020). Investigation of the STOX1 polymorphism on lumbar disc herniation. *Molecular genetics & genomic medicine*.

[5] Goker B., Aydin S. (2020). Endoscopic surgery for recurrent disc herniation after microscopic or endoscopic lumbar discectomy. *Turkish neurosurgery*.

[6] Liu C., Zhou Y. (2019). Percutaneous endoscopic lumbar discectomy and minimally invasive transforaminal lumbar interbody fusion for massive lumbar disc herniation. *Clinical Neurology and Neurosurgery*.

[7] Rogerson A., Aidlen J., Jenis L. G. (2019). Persistent radiculopathy after surgical treatment for lumbar disc herniation: causes and treatment options. *International Orthopaedics*.

[8] Wang Y., Yan Y., Zhang J. (2019). Outcomes of percutaneous endoscopic trans-articular discectomy for huge central or paracentral lumbar disc herniation. *International Orthopaedics*.

[9] World Medical Association (2013). World medical association declaration of helsinki: ethical principles for medical research involving human subjects. *JAMA*.

[10] Yüce I., Kahyaoğlu O., Mertan P., Çavuşoğlu H., Aydın Y. (2019). Analysis of clinical characteristics and surgical results of upper lumbar disc herniations. *Neurochirurgie*.

[11] Benzakour T., Igoumenou V., Mavrogenis A. F., Benzakour A. (2019). Current concepts for lumbar disc herniation. *International Orthopaedics*.

[12] Donohue D. (2020). A primary care answer to a pandemic: keeping a population of patients safe at home through chronic care management and remote patient monitoring. *American Journal of Lifestyle Medicine*.

[13] Yu X., Yang X. (2019). Remote patient management for emerging geographical areas. *Contributions to Nephrology*.

[14] Davis T. C., Hoover K. W., Keller S., Replogle W. H. (2020). Mississippi diabetes telehealth network: a collaborative approach to chronic care management. *Telemedicine and e-Health*.

[15] Walkden J. A., McCullagh P. J., Kernohan W. G. (2019). Patient and carer survey of remote vital sign telemonitoring for self-management of long-term conditions. *BMJ health & care informatics*.

[16] Paulsen R. T., Rasmussen J., Carreon L. Y., Andersen M. Ø (2020). Return to work after surgery for lumbar disc herniation, secondary analyses from a randomized controlled trial comparing supervised rehabilitation versus home exercises. *The Spine Journal: Official Journal of the North American Spine Society*.

[17] França F. J. R., Callegari B., Ramos L. A. V. (2019). Motor control training compared with transcutaneous electrical nerve stimulation in patients with disc herniation with associated radiculopathy: a randomized controlled trial. *American Journal of Physical Medicine and Rehabilitation*.

[18] Wang Q., Zhang H., Zhang J., Zhang H., Zheng H. (2019). The relationship of the shear wave elastography findings of patients with unilateral lumbar disc herniation and clinical characteristics. *BMC Musculoskeletal Disorders*.

[19] Kong L., Shang X.-F., Zhang W.-Z. (2019). Percutaneous endoscopic lumbar discectomy and microsurgical laminotomy. *Orthopäde, Der*.

[20] Goh G. S., Soh R. C. C., Yue W.-M., Guo C.-M., Tan S.-B., Chen J. L. (2020). Determination of the patient acceptable symptom state for the Japanese orthopaedic association score in patients undergoing anterior cervical discectomy and fusion for cervical spondylotic myelopathy. *The Spine Journal*.

[21] Schoenenberger A. W., Russi I., Weberndörfer B. (2020). Evaluation of comprehensive geriatric assessment in older patients undergoing pacemaker implantation. *BMC Geriatrics*.

[22] Kato S., Oshima Y., Taniguchi Y., Tanaka S., Takeshita K. (2019). Minimum clinically important difference and patient acceptable symptom state of Japanese orthopaedic association score in degenerative cervical myelopathy patients. *Spine*.

[23] Domes C. M., Schleyer A. M., McQueen J. M., Pergamit R. F., Beingessner D. M. (2017). Evaluation of appropriate venous thromboembolism prophylaxis in patients with orthopaedic trauma with symptom-driven vascular and radiographic studies. *Journal of Orthopaedic Trauma*.

[24] Goh G. S., Soh R. C. C., Yue W.-M., Guo C.-M., Tan S.-B., Chen J. L.-T. (2021). The patient acceptable symptom state for the Oswestry Disability Index following single-level lumbar fusion for degenerative spondylolisthesis. *The Spine Journal*.

[25] Yoo J. S., Patel D. S., Hrynewycz N. M., Brundage T. S., Mogilevsky F. A., Singh K. (2020). The effect of preoperative symptom duration on postoperative outcomes after minimally invasive transforaminal lumbar interbody fusion. *Clinical Spine Surgery: A Spine Publication*.

